The article "Changing the pattern of the back-muscle flexion–relaxation phenomenon through flexibility training in relatively inflexible young men" was published in 2021. Journal: PLoS One.

# Changing the pattern of the back-muscle flexion–relaxation phenomenon through flexibility training in relatively inflexible young men

**DOI:** 10.1371/journal.pone.0259619

**Published:** 2021-11-05

**Authors:** Yi-Lang Chen, Wei-Cheng Lin, Ying-Hua Liao, Yi Chen, Pei-Yu Kang

**Affiliations:** 1 Department of Industrial Engineering and Management, Ming Chi University of Technology, New Taipei, Taiwan; 2 Department of Computer Science and Information Engineering, National Taiwan University, Taipei, Taiwan; University of L’Aquila, ITALY

## Abstract

Although several studies have investigated the back-muscle flexion–relaxation phenomenon (FRP), the effect of individual flexibility on the FRP has been discussed infrequently, with very limited data on the influence of flexibility training on the FRP. This study thus examined the effect of flexibility training on the change of back-muscle FRP pattern in relatively inflexible young men. We collected and analyzed the valid data from 20 male participants (10 each with high and low flexibility included in the control and trained groups, respectively) when flexing their trunks at seven trunk flexion positions (0°–90°, in increments of 15°); their erector spinae and hamstring activation, pelvic tilt, and lumbosacral angle were then recorded. After 7 weeks of flexibility training for the low-flexibility group, no difference in flexibility was discovered between this group and the control (originally high-flexibility) group. The trunk flexion experiment was then repeated. The results showed that before the training stage, the low-flexibility group had lower erector spinae and higher hamstring activation, a larger pelvic tilt, and a smaller lumbosacral angle. By contrast, after training, the erector spinae and hamstring activation, pelvic tilt, and lumbosacral angle were significantly changed, and no intergroup differences were observed in FRP patterns. The study results suggest that flexibility training changes lumbopelvic movement and thereby reduces the degree of the back-muscle FRP when trunk flexion is performed.

## Introduction

Static upper-trunk deep flexion postures and prolonged stooping often occur in daily life and in the workplace [1, 2]. Although experts have suggested squatting to be a safer posture than stooping, field surveys have revealed that the stoop posture is considered the most efficient posture at work and most frequently adopted by workers, however, the risk of the posture to the spine was commonly ignored [3, 4].

Trunk flexion results in a heavy load on the lumbar spine owing to the torque generated by the posture [5]. When the trunk is flexed, the lumbar spine and pelvis exhibit the lumbopelvic rhythm, which involves interactions among active tissues (such as muscles and tendons), passive tissues (such as vertebrae, intervertebral discs, ligaments, and fascia), and neural control units [6]. During trunk flexion, the muscle activity of the back first increases with an increase in trunk flexion; then, the activity suddenly reduces when the trunk nearly reaches its maximum range of motion (ROM). This is termed as the back muscle flexion-relaxation phenomenon (FRP) [7] and indicates a transition of load from active lumbar tissues to passive tissues [8–10], which is part of the load-sharing synergy based on the lumbopelvic movement.

Gupta [11] investigated the relationship between the FRP and lumbopelvic movement and observed that the FRP and intense hamstring muscle activity occurred when the hip rotation and lumbar flexion were at 57% and 84%, respectively, of their maximum ROM. When the participants’ pelvis movement was restricted, the FRP may occur earlier. This observation indicated that restricting pelvic rotation results in greater lumbar flexion, causing higher tension in passive tissues and an earlier FRP during trunk flexion [12–14].

Individual flexibility also influences lumbopelvic movement and the activity of related muscles during trunk flexion. Sánchez-Zuriaga et al. [15] discovered that participants with greater lumbar flexibility had significantly less pelvic flexibility, and that lumbopelvic flexibility affected neuromuscular responses in the trunk musculature during trunk flexion–extension, leading to different load-sharing and muscle responses. The toe-touch test is a widely used flexibility measurement; during this test, the participant is required to flex their trunk when standing and to touch the ground with a fingertip [4, 16]. Hashemirad et al. [17] indicated that during trunk flexion, back muscles in individuals with superior toe-touch scores were relatively inactive at larger trunk and hip angles and were then reactivated earlier during extension. They concluded that flexibility plays a crucial role in the trunk’s muscular recruitment pattern and the strategy of the central nervous system in providing stability. This finding implies that during a deep stoop, the passive tissue loads applied in flexible individuals may be lower than those applied in less flexible people. In addition, Chen et al. [18] discovered that flexible participants exhibited a less obvious FRP than inflexible participants when performing an identical deeper trunk flexion. Hamstring flexibility is typically examined in the toe-touch test and influences the spinal posture when trunk flexion is performed. However, studies have examined the effects of hamstring flexibility on the FRP only by evaluating the various flexibility levels of participants [4, 14, 19].

Several studies have employed various stretching programs for increasing hamstring flexibility [20, 21] and have identified significant improvements [16, 22–24]. Muyor et al. [16] had participants perform three hamstring stretching sessions each week, and they demonstrated significant increases in toe-touch test scores after 12 weeks. Battaglia et al. [25] applied the flexibility training program of Muyor et al. [16] and randomly recruited 37 participants for 8 weeks of intensive flexibility training; and the trained group had a significantly improved spinal curve, sacrum or hip rotation, and thoracic flexion. On the basis of all these study findings, the present study examined whether flexibility can be acquired through training (based on the study results of Muyor et al. [16]) and consequently whether the FRP pattern can be changed. We hypothesized that before training, the FRP pattern would differ between the groups with initially low and high flexibility, and that after training, no differences would exist in the FRP between the two groups. If this hypothesis can be confirmed, trained flexibility can be an effective strategy for changing back-muscle FRP patterns.

## Methods

### Participants

This study originally recruited 22 male university students aged 18–23 years as participants. Recruitment was through announcements on the bulletin board of Ming Chi University of Technology (New Taipei, Taiwan) during January 1–20, 2019. The volunteers were then interviewed and informed of the details of the test procedure. All participants were right handed, and none had a history of musculoskeletal injury or lower back pain. All participants agreed to avoid staying up late or engaging in strenuous activity throughout the experimental period. Participants were familiarized with the test procedures and were paid for their participation. The experimental procedures were approved by the National Taiwan University (NTU-REC NO. 201712EM014), and all participants provided written consent before the experiment.

Participants were divided into groups with low (n = 12) and high (n = 10) flexibility on the basis of the toe-touch flexibility test, which was adopted from the studies of Shin et al. [4] and Ayala et al. [26]. During the test, participants flexed their trunk, keeping their knees straight, and attempted to touch and overreach the floor baseline with their fingertips. Participants who touched the floor and reached 3 cm below the floor baseline were included in the high-flexibility group, whereas those who failed to reach the floor baseline more than 3 cm were included in the low-flexibility group [14, 18]. Among the 12 participants in the low flexibility group, two participants failed to finish the stretching program due to time schedule and were thus excluded from the data analyses. Table 1 presents the anthropometric data of the participants in each group (n = 10 for each). The independent *t* test revealed no significant differences between the groups in any variable other than flexibility. The mean (standard deviation) flexibility score of the high- and low-flexibility groups was 7.6 (3.2) and −7.2 (4.1) cm, respectively. The average difference between the two groups was 14.8 cm (p < .001).

**Table 1:** Demographic data of the participants in the study (n = 10 for each group).

Variables	Flexible (control) group		Inflexible (trained) group		Differences
	Mean (SD)	Range	Mean (SD)	Range	
Age (years)	19.8(1.4)	18–23	19.3(1.2)	18–21	0.5
Height (cm)	173.2(3.2)	170–179	174.9(3.7)	168–179	-1.7
Weight (kg)	65.6(8.0)	56–80	67.4(8.6)	55–80	-1.8
Acromial height (cm)	143.2(3.4)	138.7–150.4	143.4(3.4)	136.5–147.6	-0.2
Knuckle height (cm)	74.3(3.5)	65.7–77.9	76.2(3.4)	71.4–82.6	-1.9
Hip height (cm)	86.5(2.3)	82.6–89.4	89.0(5.5)	81.2–101.5	-2.5
Knee height (cm)	48.3(2.1)	45.6–51.2	49.2(2.4)	45–52.5	-0.9
Flexibility (cm)					
before training stage	7.6(3.2)	4.0–18.0	-7.2(4.1)	(-10.4)-(-3.2)	14.8*
after training stage	7.5(3.4)	3.7–18.9	7.4(3.6)	3.0–8.9	0.1

* significantly different between two groups using an independent *t* test (p < .001).

### Flexibility training

Twelve young male students participated in the flexibility training program as adopted by Muyor et al. [16]. Consequently, ten participants in the trained group successfully completed the program and two were excluded because they missed too many training sessions (> 2 days). The stretching program was continually monitored and recorded by an investigator, who was well-trained with the stretching protocols. The hamstrings were stretched with hip in flexion and knee in extension, with the spine maintained in a normal position, and with participants in orthostatic, sitting, and supine positions (Fig 1) [16]. In all stretching exercises, stretched positions were assumed gently and slowly until the endpoint of range. Once this position was achieved, participants held it for 20 s. The experimenter instructed them to feel a strain on the hamstring muscles without feeling pain. By contrast, participants in the control group did not participate in the program or any other intensive physical activity.

**Fig 1:** Schematic of stretching postures adopted in the training stage.

The experimental (trained) group participated in a program three times a week (Monday, Wednesday, and Friday, between 17:10 and 17:40 hours, 15 min per day) after the students’ classes and scheduled for a period of 6 to 10 weeks depending on results [25]. It indicated that the training will be stopped once no difference in the flexibility was observed between the two groups. If a participant missed a training session, he made up for the missed session on the next day. Any participant who missed more than 2 days of training was excluded from data analysis. All participants were instructed not to participate in any other intensive physical activity and not to alter their daily habits during the study. The toe-touch test was performed and analyzed before and after the stretching program for the trained (n = 10) and control groups (n = 10).

### Lumbar and pelvic posture measurements

Pelvic tilt and spinal curvature (i.e., lumbosacral angle [LSA]) were measured while participants stood upright and flexed their trunk to 90° in increments of 15°; this angle was formed by the line linking the acromial shelf and hip to the vertical. Before data collection, we attached five adhesive reflective markers to specific joints (i.e., the acromial shelf, the caudal-most point of the iliac crest, hip, knee, and ankle) and used two stick markers on specific skin areas (i.e., first lumbar and first sacral spinous processes; Fig 2). We measured the pelvic tilt in accordance with the method of Chen and Lee [27] and the external LSA (formed by S1 and L1) that was subsequently used as a reference to calculate the internal LSA by using the prediction models also developed by Chen and Lee for predicting the vertebral inclination of the lumbar spine:

$${IL}_{1}=0.9882\times {SL}_{1}+3.6274\;\left(R^{2}=0.968\right)$$

$${IS}_{1}=0.7339\times {SS}_{1}+29.6776\;\left(R^{2}=0.916\right)$$

Herein, SL1 and SS1 represent the respective angles of the external markers L1 and S1 (Fig 2), and IL1 and IS1 are the internal angles. The internal LSA was obtained by determining the angle between IL1 and IS1.

**Fig 2:** Schematic of testing posture, body angles, and marker and sticker positions.

### Electromyography

An electromyography (EMG) device, TeleMyo 2400 (Noraxon, Scottsdale, AZ, USA), was used to analyze the two muscle groups (erector spinae and hamstring) on each participant’s dominant side. The EMG testing procedure (including skin preparation, electrode location, placement, and fixation), data acquisition and processing were performed mainly according to the recommendations by the Surface Electromyography for the Noninvasive Assessment of Muscles (SENIAM) [28–30]. We placed pairs of Ag/AgCl surface electrodes (lead-off area, 10 × 10 mm2; center-to-center electrode distance, approximately 20 mm) parallel to the muscles. Before electrode attachment to the skin, the area was shaved and cleaned with alcohol. Bipolar surface electrodes were attached to the skin with adhesive tape to prevent artifacts, as suggested by SENIAM [28]. For the erector spinae and hamstring muscles, the electrodes were placed at 2 finger width lateral from the spinal process of L1 and 50% on the line between the ischial tuberosity and the medial epycondyle of the tibia, respectively.

Before EMG recording, participants performed standardized muscle-specific maximal voluntary contractions (MVCs) to normalize signals measured for each trunk posture trial. MVC testing was performed as described by Vera-Garcia et al. [31], and the following MVC techniques were used for the muscle groups: for the erector spinae, participants attempted to extend the lower trunk and the hips against manual resistance in a prone position with the torso on a bench and the legs horizontally cantilevered over the end of the bench [31]; for the hamstring, participants were in a prone position with their knees at 30° flexion with maximal effort against manual resistance [32]. Participants were given strong verbal encouragement during each MVC measurement. For all the muscles tested, participants were instructed to perform the MVC three times and to hold for at least 5 s each, with a 3-min rest interval between contractions. The highest value in these three measures was used as the MVC value for further analysis. Electrical signals collected from both MVC tests and testing trials were filtered through the high and low frequencies of an analog band-pass filter (20–600 Hz) before they were sampled (1200 Hz) [29, 30]. Sampled signals were then completely rectified and processed to produce integrated EMG (IEMG) data. A normalization procedure was then performed to compare IEMG data from the experimental trial with the MVC IEMG data with an identical interval of 5 s. All muscle activation values are presented as percentages of the IEMG data of the MVC.

### Experimental design and procedure

Before beginning the flexibility training program, the FRP experiment was performed with the two flexibility groups. We recorded muscle activation, pelvic tilt, and the LSA at various trunk angles for all participants. The experimental setting was based on that of Chen et al. [18]. The trunk flexion angles were 0°–90° in increments of 15°. During the experiment, participants were required to flex their trunk from an upright position to the six specific trunk angles and keep their knees straight with their hands positioned over their navel area (Fig 2). Once participants had bent their trunk to the requested angle, they sustained the posture for 10 s. The motion and EMG data obtained for the final 5 s of each position were used for analyses. We employed a trigger signal to begin the collection of both motion and EMG data to ensure synchronization. A minimal rest period of 5 min was allowed between successive trials to prevent muscle fatigue, and each participant was tested for less than 1.5 h. All participants performed each test combination two times for reliability examination, and mean values were considered for further analysis. Subsequently, pelvic tilt, LSA, and static EMG data (of two muscle groups) were recorded for each participant from 14 test combinations (7 trunk angles × 2 repetitions). To prevent experimental errors, the 14 combinations were randomly arranged for each participant.

During the test, a MacReflex motion analysis system (Qualisys, Göteborg, Sweden) was positioned approximately 5 m to the left lateral side of the participant and perpendicular to the participant’s sagittal plane and recorded the 2D marker positions (resolution = 1:30,000 in the camera field of view at 120 Hz and low-pass filtered at 6 Hz). The experimenter verified that the participant’s trunk line (i.e., the connection between the shoulder and hip markers) matched a preset line in the feedback monitor of the motion analysis system to ensure that the torso flexion angle of each participant was in the desired position.

After completion of the flexibility training program, the FRP experiment was repeated with the two flexibility groups. The posture and EMG data acquired before and after training were then compared.

### Statistical analysis

The participants’ muscle activity, pelvic tilt, and LSA were analyzed using SPSS 22.0; the significance level was set at α = .05. In this study, Pearson product-moment correlation (r) was used to explore the repeat reliability of the EMG and lumbopelvic measurements, and the independent *t* test was used to identify any difference in anthropometry and flexibility (before and after training) data between the two groups. Subsequently, a 2-way analysis of variance (ANOVA) was performed to determine how flexibility training influenced muscle activity, pelvic tilt, and LSA. The independent variables were flexibility group (4 groups comprised of 2 flexibility levels and 2 training stage) and trunk flexion (7 trunk positions). Each participant was considered a block and Duncan’s multiple range test was used for *post hoc* comparisons.

## Results

### Flexibility training results

In the study, 10 participants completed the flexibility training program. After 7 weeks of flexibility training, the mean (standard deviation) flexibility of the trained group increased from −7.2 (4.1) to 7.4 (3.6) cm, an improvement of 14.6 cm. The average flexibility score was nonsignificantly different from that of the control group (7.5 cm, as shown in Table 1), indicating that hamstring flexibility was improved by continual regular stretching exercises. Because no difference in flexibility was observed between the two groups, the training was stopped for the training group, and an FRP experiment was performed to clarify the effect of the flexibility training on the FRP pattern.

### Two-way ANOVA results

The measurement repeatability of each muscle activation, pelvic tilt, and LSA for all participants was higher than 0.815 (all p < .05), indicating satisfactory consistency. Body posture and muscle activation data for each trunk position in the two flexibility groups before and after training are presented as (S1 Table). Table 2 shows the two-way ANOVA results. The trunk angle and flexibility variable (high and low flexibility, before and after training; i.e., four combined variables) had a significant effect on all responses (all p < .01), and the two-factor interactions were nonsignificant. Table 3 shows that when the trunk was flexed from the erect position, the erector spinae and hamstring were increasingly activated, but when the erector spinae and hamstring reached their maximum activation at 45° and 60° of trunk flexion, respectively; muscle activation decreased as the angle increased to 90°, indicating that the FRP had occurred in both muscle groups. When the flexibility variable was averaged across the trunk angle, the results revealed that the untrained low-flexibility group exhibited less erector spinae and greater hamstring activation than did the trained and originally flexible groups (Table 4). The result is also evident from Figs 3 and 4. Table 5 shows that both the pelvic tilt and LSA increased with an increase in the trunk angle and were lowest when the trunk position was 90°. Furthermore, Table 6 shows that the low-flexibility group had significantly greater pelvic tilt and lower LSA before training than did the others (Figs 5 and 6).

**Fig 3:** Changes in erector spinae activation (mean and standard deviation) in the two participant groups before and after flexibility training stage (HiFx: High flexibility; LoFx: Low flexibility).

**Fig 4:** Changes in hamstring activation (mean and standard deviation) in the two participant groups before and after flexibility training stage (HiFx: High flexibility; LoFx: Low flexibility).

**Fig 5:** Changes in pelvic tilt (mean and standard deviation) in the two participant groups before and after flexibility training stage (HiFx: High flexibility; LoFx: Low flexibility).

**Fig 6:** Changes in lumbosacral angle (mean and standard deviation) in the two participant groups before and after flexibility training stage (HiFx: High flexibility; LoFx: Low flexibility).

**Table 2:** Two-way ANOVA results of the measurements.

Variables	Measurements	DF	SS	MS	F	*p*	Power
Trunk angle (TA)	Erector spinae	6	5745	957	130.0	<0.001	1.000
	Hamstring	6	2887	481	29.2	<0.001	1.000
	Pelvic tilt	6	26184	4364	146.4	<0.001	1.000
	Lumbosacral angle	6	166096	27683	689.5	<0.001	1.000
Flexibility group (FG)	Erector spinae	3	145	48	6.5	<0.001	0.970
	Hamstring	3	373	124	7.5	<0.001	0.986
	Pelvic tilt	3	487	162	5.4	0.001	0.935
	Lumbosacral angle	3	2020	674	16.8	<0.001	1.000
TA ×FG	Erector spinae	18	109	6	0.8	0.674	0.595
	Hamstring	18	133	7	0.5	0.976	0.313
	Pelvic tilt	18	230	13	0.4	0.981	0.300
	Lumbosacral angle	18	203	11	0.3	0.999	0.195

**Table 3:** Muscle activation of Duncan groups for varying trunk angles.

Trunk angles (°)	N	Erector spinae (%MVC)	Duncan groups	Hamstring (%MVC)	Duncan groups
0	40	4.2 (0.8)	A	1.5 (0.4)	A
15	40	10.4 (2.0)	B	6.9 (3.7)	B
30	40	14.8 (2.8)	C	9.8 (4.2)	CD
45	40	15.5 (2.9)	C	11.3 (4.4)	D
60	40	10.1 (5.4)	B	11.6 (5.1)	D
75	40	5.0 (1.7)	A	10.8 (4.2)	CD
90	40	4.0 (1.3)	A	9.1 (4.6)	C

**Table 4:** Muscle activation of Duncan groups for varying flexibility and training combinations.

Groups	N	Erector spinae (%MVC)	Duncan groups	Hamstring (%MVC)	Duncan groups
HiFx_before training stage	70	9.4 (2.7)	A	8.1 (2.7)	B
HiFx_after training stage	70	9.6 (2.3)	A	7.6 (2.6)	B
LoFx_before training stage	70	8.0 (1.7)	B	10.5 (5.4)	A
LoFx_after training stage	70	9.5 (2.0)	A	8.6 (3.0)	B

Notes: HiFx, high-flexibility; LoFx, low-flexibility

**Table 5:** Pelvic tilt and lumbosacral angle of Duncan groups for varying trunk angles.

Trunk angles (°)	N	Pelvic tilt (°)	Duncan groups	Lumbosacral angle (°)	Duncan groups
0	40	53.1 (4.2)	A	50.3 (4.9)	A
15	40	49.8 (4.4)	B	38.1 (6.3)	B
30	40	45.4 (5.0)	C	22.0 (6.8)	C
45	40	41.4 (6.3)	D	7.6 (8.5)	D
60	40	37.5 (6.5)	E	-3.9 (7.7)	E
75	40	31.1 (6.2)	F	-14.1 (6.0)	F
90	40	23.5 (5.1)	G	-20.6 (5.5)	G

**Table 6:** Pelvic tilt and lumbosacral angle of Duncan groups for varying flexibility and training combinations.

Groups	N	Pelvic tilt (°)	Duncan groups	Lumbosacral angle (°)	Duncan groups
HiFx_before training stage	70	39.2 (10.6)	B	14.3 (6.3)	A
HiFx_after training stage	70	39.8 (11.5)	B	11.9 (5.3)	A
LoFx_before training stage	70	42.5 (10.7)	A	6.8 (5.5)	B
LoFx_after training stage	70	39.5 (11.3)	B	12.4 (6.0)	A

Notes: HiFx, high-flexibility; LoFx, low-flexibility

## Discussion

In this study, 10 participants with low toe-touch scores (trained group) were compared with 10 participants with high toe-touch scores (control group), and their FRP patterns before and after training were analyzed. Before training, a difference in the FRP was observed between the low-and high-flexibility groups. The low-flexibility group was then trained through a flexibility program, and after 7 weeks of flexibility training, their toe-touch scores were nonsignificantly different from those of the high-flexibility group; the FRP experiment was then repeated for comparison. This study showed that increased flexibility changed the participants’ FRP patterns; that is, the patterns of the groups became indistinguishable, showing that the flexibility training reduced the degree of the FRP, but without significantly affecting the time of FRP occurrence. This result verified the study hypothesis.

This study applied the flexibility training method proposed by Muyor et al. [16], and it was intensified by increasing the training duration (i.e., 15 min per day). After the 7-week training, the toe-touch scores were 7.5 and 7.4 cm for the control (i.e., originally flexible) and trained groups, respectively, indicating no significant intergroup difference. This study confirmed that increased flexibility reduces the degree of the FRP. Previous research has determined that when the trunk is flexed, flexible people exhibit a milder FRP, regardless of the standing posture in both sexes [4, 18] and the sitting posture in men [33]. The current study demonstrated that the flexible group of men exhibited a similar effect of a smaller FRP upon standing. In accordance with previously conducted experiments, this study recruited participants with different flexibility levels to perform the FRP experiment, and the results were consistent with those of previous studies [4, 18]. Participants with different levels of flexibility exhibited dissimilar FRP patterns; that is, the less flexible participants exhibited a more obvious FRP (Fig 3), larger pelvic tilt (Fig 4), and smaller LSA (Fig 5). These findings indicated that when the trunk is flexed to an assigned position, pelvis rotation is limited because of the reduced extensibility of the hamstrings in the low-flexibility group, thereby necessitating more lumbar flexion. Nevertheless, the hamstring activation in the participants with low flexibility indicated greater muscle contractions (Fig 3).

In this study, the toe-touch test was used to distinguish between participants with high and low flexibility; this test assesses the extension of the back and hamstring muscles simultaneously. Hashemirad et al. [17] identified that during trunk flexion, the erector spinae muscles in individuals with higher toe-touch scores were relatively inactive for larger trunk and hip angles, implying that flexibility may play a crucial role in the trunk’s muscular recruitment pattern. The present study revealed that the high-flexibility group exhibited higher erector spinae and lower hamstring muscle activation, which could have caused the pelvis to fully rotate forward and offer the advantage of spinal stability during flexion. Sihvonen [34] observed that the hamstring produces a similar FRP, but the FRP occurs later than that of the erector spinae. In addition to the FRP caused by the elongation of the erector spinae, an FRP was generated through the elongation of the hamstring that was related to pelvic movement and involved in trunk flexion.

This study identified that the FRP of the hamstring was delayed compared with that of the erector spinae, which occurred at trunk positions between 60° and 75°. Gupta [11] indicated that when the FRP occurred, all their participants exhibited greater hamstring muscle activation during trunk flexion. In this study, the FRP in the back muscles occurred at trunk positions between 45° and 60°, and the activity of the hamstrings was observed to be highest at this moment. Furthermore, Solomonow et al. [35] observed that the FRP of 49 participants occurred at approximately 45°–50° trunk positions, which is consistent with the results of the present study, whereas Chen et al. [18] observed the FRP to occur at approximately 60°. Eungpinichpong et al. [13] identified greater lumbar flexion and smaller back-muscle activation when a person was wearing jeans, which limits lumbopelvic movement. The effect of jeans on the FRP appears to be similar to that of low flexibility in the low-flexibility group of our study.

In this study, the flexibility training program probably extended the range of trunk movement as well as the extensibility of the hamstrings. Because of the increase in flexibility, the mechanism of lumbopelvic movement changed; therefore, the degree of the FRP was reduced. This observation implies that flexibility acquired by training can also reduce the degree of the FRP, which may reduce the force on passive tissues close to the lumbar region when an identical deep trunk flexion is performed. Gajdosik et al. [36] and López-Miñarro and Alacid [37] identified different patterns of spinal and pelvic postures in men on the basis of their hamstring flexibility differences. Individuals with higher hamstring flexibility exhibited greater anterior pelvic inclination. This finding could be the evidence needed to explain the result of our study.

## Conclusion

This study successfully trained 10 participants (trained group) with low flexibility for 7 weeks to improve the flexibility. Another 10 participants with high flexibility were recruited as the control group. Results showed that, although a difference was found between the two groups’ FRP patterns before training, no FRP difference was discovered after the training. Flexibility training may extend the ROM of trunk movement and decrease the pelvis tilt during trunk flexion; it may thus reduce the degree of the FRP. Previous studies have shown that flexible people exhibit the less obvious FRP than relatively inflexible individuals; this study further verifies that flexibility training exerts an effect through improvement in the lumbopelvic movement. These findings indicate that the stretching protocols adopted in the study may be practically valuable for people when work or daily activity involve a deep trunk flexion. However, the participants recruited from the study were young men, whether the results are applicable to older people or on-site workers needs further investigation.

## Supporting information

S1 Table Body posture and muscle activation data for each trunk position in the two flexibility groups before and after training. (XLSX)
